# Myogenic regulatory factors are key players in determining muscle mass and meat quality in Jeju native and Berkshire pigs

**DOI:** 10.1002/vms3.418

**Published:** 2020-12-29

**Authors:** Kyoungho Kim, Dahye Kim, Yunhui Min, DongKee Jeong, Young‐Ok Son, Kyoungtag Do

**Affiliations:** ^1^ Department of Animal Biotechnology Faculty of Biotechnology College of Applied Life Sciences Jeju National University Jeju‐si Jeju Special Self‐Governing Province Republic of Korea; ^2^ Livestock Division Jeju‐si Jeju Special Self‐Governing Province Republic of Korea; ^3^ Interdisciplinary Graduate Program in Advanced Convergence Technology and Science Jeju National University Jeju‐si Jeju Special Self‐Governing Province Republic of Korea; ^4^ Bio‐Health Materials Core‐Facility Center Jeju National University Jeju‐si Jeju Special Self‐Governing Province Republic of Korea; ^5^ Practical Translational Research Center Jeju National University Jeju‐si Jeju Special Self‐Governing Province Republic of Korea

**Keywords:** Berkshire, Jeju native pig, MyBPH, MyoD, myogenic regulatory factor, Pax7

## Abstract

**Background:**

Meat from Jeju native pigs (JNPs) is highly popular among Korean consumers; however, the production efficiency is limited due to the low adult body weight. In contrast, the Berkshire breed, which has a genetic background closely related to Asian native pigs, gains weight more efficiently.

**Objectives:**

This study focused on the differential expression of genes related to muscle growth in postnatal myogenesis between Berkshire and JNPs, specifically the myogenic regulatory factor (MRF) genes (MyoD, Pax7, Myf5, Myf6 and MyBPH). The MRF family is primarily involved in the proliferation and development of muscle.

**Methods:**

Qualitative reverse transcription‐polymerase chain reaction and western blot analyses revealed that expression of MyoD and Pax7 was significantly higher in Berkshire pigs than in JNPs. In addition, co‐expression of MyoD and Pax7 was observed in myotubes formed in cultured C2C12 cells. ToppCluster was used to elucidate the relationship between biological processes of the MRFs and muscle‐related signalling pathways.

**Results:**

MyoD and Pax7 are factors essential for the activation of satellite cell during myogenesis. However, the mRNA and protein levels of MyBPH (which is responsible for meat quality, e.g. water content, colour and tenderness) are significantly higher in both 1‐day‐old piglets and adult JNPs than in Berkshire pigs.

**Conclusions:**

This study provides a genetic understanding of myogenesis in the postnatal and adult stages of Berkshire pigs and JNPs. Moreover, these results will help identify marker genes related to muscle mass, growth performance and meat quality in indigenous Korean pig breeds.

## Graphical abstract

High expression of MyoD and Pax7 are strictly relative muscle mass with the activation of satellite cells in Berkshire breed, whereas high expression of MyBPH involves meat quality in JNPs breed.

## 1 INTRODUCTION

The skeletal muscle occupies 20%–50% of the total body mass and is one of the primary tissues involved in meat production (Qazi et al., 2015; Wu et al., 2013). In the last few decades, several studies have evaluated genes to understand the underlying mechanisms of the proliferation and development of muscle tissue in pigs (Liu et al., 2012). Several factors are responsible for postnatal skeletal muscle growth. First, myofibres and multinucleated fibres act as the functional unit of skeletal muscle and are generated by the fusion of myoblasts to form multinucleated tubes (Järvinen et al., 2007; Järvinen et al., 2005; Qazi et al., 2015). Second, multipotent stem cells, known as satellite cells, are believed to contribute to the growth of muscle fibres (Carnes & Pins, 2020; Qazi et al., 2015). The satellite cells comprise only 2%–7% of the total myonuclei (Rudnicki et al., 2008). Satellite stem cells express Pax7, while satellite myogenic cells also activate myogenic factor‐5 (Myf5) and myogenic determination factor (MyoD0 (Rudnicki et al., 2008). Therefore, Pax7, Myf5 and MyoD activity are closely related to satellite cell activation (Lepper et al., 2011; von Maltzahn et al., 2013; Murphy et al., 2011; Sambasivan et al., 2011).

Jeju Island in South Korea has unique subtropical climatic conditions, with characteristic native fauna and flora. For example, Jeju native pigs (JNPs) are more tender and juicy, with more marbling than the meat of other foreign pig breeds (Cho et al., 2011; Kim & Kim, 2018). Consequently, the meat of JNPs has gained popularity among Chinese, Japanese, and Korean consumers. Therefore, JNPs are one of the most expensive pork breeds in Asian countries (Kim et al., 2013). Despite the disease‐resistant traits of JNPs, their slow growth rate, low feed consumption and low production efficiency are significant obstacles in JNP breeding (Sodhi et al., 2014). To overcome these issues, JNPs were crossbred with Berkshire pigs, as these are considered a breed suitable for meat production. Thus, practical breeding of JNPs was achieved by crossbreeding with Berkshire pigs (Hur et al., 2013; B.‐W. Kim et al., 2011). Crossbred pigs of JNPs and Berkshire pigs exhibited improved meat quality; thus, this meat is highly popular among Korean consumers. Currently, crossbreeding has become a unique aspect of the pork industry in Asian countries. Thus, JNPs and Berkshire pigs are often used in studies aiming to improve meat quality and muscle growth rates in the pig industry (Yu et al., 2013). In order to elucidate the molecular mechanisms underlying muscle growth and meat quality or palatability, comparative analysis of genes among various breeds has been performed. For example, identification of differentially expressed genes in the *longissimus dorsi* muscle was performed in Wei and Yorkshire pigs (Xu et al., 2018), JNPs and miniature pigs (Ghosh et al., 2019), Northeast Min pig (NM) and Changbaishan wild boar (CW) (Xu et al., 2019), and between the Chinese indigenous Min pig and the Large White pig (Liu et al., 2017).

Usually, food scientists consider the size, number, area and density of muscle fibres as the main traits defining meat quality (Ryu & Kim, 2006); however, the Rika Ito group recently reported a correlation between the growth of muscle mass and the number of myotubes (Ito et al., 2018). Satellite cells are also involved in the growth and regeneration of skeletal muscle during postnatal fertilization (Ropka‐Molik et al., 2011). Satellite cells are surrounded by myotubes, which play a significant role in muscle proliferation and hypertrophy (Zammit et al., 2006). Muscle‐specific genes are regulated by the basic helix–loop–helix (bHLH) transcription factors involved in muscle proliferation, development and growth (Te Pas et al., 2007). Myogenic regulatory factors (MRFs) are members of the bHLH family. MRFs are composed of MyoD, Myf5, myogenic factor‐6 (Myf6) and myogenin. Furthermore, MyoD is involved in the differentiation of skeletal muscle cells and satellite cell activity associated with paired box transcription factor‐7 (Pax7) (Mesires & Doumit, 2002).

A study on porcine muscle reported that the *Pax7* gene induces the self‐renewal of satellite cells and influences the dynamic stages in muscle growth during postnatal fertilization (Patruno et al., 2008). Myosin fibres in the striated muscle consist of a group of myosin‐binding proteins (MyBPs) that exist in two forms: MyBP‐C and MyBP‐H (Gruen & Gautel, 1999). It has been reported that muscle fibre composition is correlated with muscle mass and body weight (Ryu & Kim, 2006). Myf6 is known as the bHLH transcription factor and regulates the differentiation of muscle fibres (Wyszyńska‐Koko & Kurył, 2004). High expression of Myf6 in the non‐fatty, dry skeletal muscle of adult pigs has been reported (Lowe et al., 1998; Te Pas et al., 2007).

Moreover, muscle growth retardation has been shown to be triggered by the inactivation of the Myf6 protein (Hinits et al., 2007). Clearly, *Myf6* is one of the genes that affects skeletal growth and quality‐related traits in adult pigs (Buonanno et al., 1992; Maak et al., 2006). However, which genes are associated with traits related to pork (meat) weight, muscle fibre properties and pork quality is not fully understood.

JNPs have been crossbred with Berkshire pigs for decades to improve meat quality; however, there are only a few studies related to muscle fibre properties in crossbred JNPs. Therefore, the aims of this study were to (1) identify candidate genes related to muscle growth based on the transcriptomic analysis of the *longissimus dorsi* muscle tissue of JNPs and Berkshire pigs, and (2) elucidate the molecular mechanisms of genes related to muscle growth by their biological functions and mechanisms. This study is expected to be a cornerstone of breed improvement programmes for JNPs and other native breeds.

## 2 MATERIALS AND METHODS

### 2.1 Animals and sample preparation

This study was conducted in compliance with the regulations of the Animal Experimental Ethics Committee of Jeju National University (No.: 2013–0009). Ten female, 1‐day‐old piglets and adult pigs (5 months old) were selected from the JNP and Berkshire pig breeds. The experimental cages were maintained at 25 ± 1°C, with temperature controlled by a heat lamp. The lamp was turned on for 10 hr from 8 a.m. to 6 p.m., and was switched off for the remaining 14 hr. Each piglet was equipped with a feeder and a water supply nipple. Water and food were provided ad libitum. One‐day‐old piglets and adult pigs (5 months old) were slaughtered according to the standard protocols of Jeju National University. The *longissimus dorsi* muscle between the 12th and 13th rib spaces was collected immediately after slaughter. Muscle samples were rapidly frozen on dry ice and stored in a −80°C freezer until RNA or protein extraction.

### 2.2 Total RNA and protein extraction

Total RNA was extracted with TRIzol™ (Invitrogen, USA) from frozen muscle tissue (120 mg) of 1‐day‐old piglets and adult pigs. After adding 400 µl of chloroform to the tissue stored in TRIzol™, the samples were mixed well and homogenized. Isopropanol (Junsei Chemical Co. Ltd., Japan) was immediately added to the homogenized tissue for RNA precipitation. After this, the pellet was washed with 1 ml 75% ethanol. The extracted RNA samples were stored at −80°C until further analysis. The RNase‐free DNase set (Qiagen, Hilden, Germany) was used to remove DNA from the extracted RNA sample using the RNeasy Mini kit (Qiagen). RNA quality was determined on a Bioanalyzer 2,100 using RNA 6,000 Nano Labchips and by automated capillary electrophoresis (Agilent Technologies Ireland, Dublin, Ireland). RNA quality was determined based on the 28/18 s ratio of 1.8, 2.0, and a RIN (RNA integrity number) value of ≥ 8.0. Total protein was extracted from the homogeniZed tissue using a radioimmunoprecipitation assay (RIPA) buffer. The protein concentration was measured using the Pierce™ BCA Protein Assay kit (Thermo Scientific, USA) on a Bio‐Rad Micro‐plate Reader (Model‐680; Bio‐Rad, USA).

### 2.3 Quantitative Real‐time polymerase chain reaction (QRT‐PCR)

The qRT‐PCR primers were prepared using the Primer‐3 program (Rozen & Skaletsky, 2000); details of the primer sequences are provided in Table 1. The Step‐One Real‐Time PCR system (Applied Biosystems) was used to check the mRNA transcript levels of *MyoD*, *Pax7*, *MyBPH*, *Myf5* and *Myf6* in JNPs and Berkshire pigs. The transcript levels of the target genes were determined using EvaGreen dye reagent (Biotium, USA). The PCR experiments were conducted in triplicate for each sample, under the following conditions: 98°C for 5 min, followed by 40 cycles of PCR; one PCR cycle consisted of 15 s at 95°C and 60 s at 60°C. The efficiency of qRT‐PCR was confirmed using the standard curve method, and the housekeeping gene *β‐actin* was used to correct the transcript expression of the target genes (Wang et al., 2006). The mRNA expression levels were compared and quantified using the two delta CT method (Livak & Schmittgen, 2001), and the relative expression was used as the result (Erkens et al., 2006; Van Poucke et al., 2001).

**TABLE 1:** List of primers used for quantitative real‐time PCR analysis of the relative quantity of transcripts in 1‐day‐old piglets and adult pigs of the Berkshire and Jeju native pig breeds

Gene Name	Primer sequences (5′−3′)	T_m_	Product size	Gene bank ID
*MyoD*	F: TGCAAACGCAAGACCACTAA R: GCTGATTCGGGTTGCTAGAC	55 °C	127	NM_001002824.1
*Pax7*	F: GGCAGAGGATCTTGGAGACA R: TGGGTGGGGTTTTCATCAAT	55 °C	144	AY653213.1
*Myf6*	F: ATCTTGAGGGTGCGGATTTC R: CAATGTTTGTCCCTCCTTCCT	62 °C	108	XM_003481764
*Myf5*	F: CCGACACAGCTTGTGGAATA R: GCCAATCAACTGATGGCTTT	55 °C	128	XM_001924362.2
*MyBPH*	F: AGTGCAGAAGGCAGACAAA R: AAGACCCGGAAGGAGTAAGA	62 °C	117	NC_010451
*β‐actin*	F: GACATCCGCAAGGACCTCTA R: ACACGGAGTACTTGCGCTCT	60 °C	157	XM_003124280

Note

Direction: F means forward, and R means reverse

### 2.4 Western blotting

Proteins were diluted 1:1 with dissociation buffer and boiled at 100°C for 10 min; samples were then analysed by electrophoresis on a 12% SDS–PAGE gel. The separated proteins were transferred onto nitrocellulose membranes using Mini‐Protean II (BioRad, Richmond, CA, USA). The membrane (Invitrogen) was transferred into a transfer buffer (12 mM Tris, 96 mM glycine, and 20% methanol; pH 8.3) for 1 hr 30 min. The membrane was then blocked with TBS containing 5% skim milk at room temperature for 1 hr and washed three times with 0.05% TBST for 10 min. Subsequently, the membrane was incubated with diluted antibodies in 3% BSA overnight at 4°C, washed three times with TBST for 10 min, and reacted with diluted secondary antibodies in 5% skim milk at room temperature for 1 hr; the antibodies used are shown in Table 2. The membrane was washed three times with TBST for 10 min and then developed using a substrate. A luminescent image analyser (LAS‐4000 mini) was used to identify specific expression bands.

**TABLE 2:** List of primary and secondary antibodies used in the expression analysis of proteins isolated from the *longissimus dorsi* muscles of 1‐day‐old piglets and adult pigs of the Berkshire and Jeju native pig breeds

Protein	Primary Antibody*	Secondary Antibody*
MyoD	Rabbit polyclonal 1:3,000 (Solarbio #K106490P)	Goat anti‐rabbit, 1:10,000 (Santa Cruz SC−2004)
Pax7	Rabbit polyclonal 1:500 (Solarbio #K002662P)	Goat anti‐rabbit, 1:10,000 (Santa Cruz SC−2004)
Myf6	Mouse monoclonal 1:200 (Santa Cruz SC−514379)	Goat anti‐mouse, 1:10,000 (Santa Cruz SC−2005)
Myf5	Mouse monoclonal 1:200 (Santa Cruz SC−518039)	Goat anti‐mouse, 1:10,000 (Santa Cruz SC−2005)
MyBPH	Mouse monoclonal 1:400 (Thermo Fisher Scienfific MA5−26185)	Goat anti‐mouse, 1:10,000 (Santa Cruz SC−2005)
β‐actin	Mouse monoclonal 1:3,000 (Solarbio #K200058M)	Goat anti‐mouse, 1:10,000 (Santa Cruz SC−2005)

### 2.5 C2C12 cell line culture

An immortalized mouse myoblast cell line (C2C12) was cultured in Dulbecco's Modified Eagle Medium (DMEM) with 20% foetal bovine serum (FBS), 100 unit/mL penicillin, 100 µg/ml streptomycin, and 100 µg/ml gentamycin. To induce differentiation into myotubes, the medium was replaced with DMEM containing 2% horse serum (HS; GIBCO^TM^, NZ).

### 2.6 Immunocytochemical analysis

C2C12 cells were seeded at a density of 1 × 10^5^ cells/well on coverslips in a 24‐well culture plate. Cells were cultured overnight, the medium was replaced with differentiation medium, and culture continued for 24 hr. Cells grown on coverslips were fixed in 4% paraformaldehyde for 30 min and washed with PBS. The cells were then treated with 0.1% Triton X‐100 (pH 7) for 10 min at room temperature. Fixed cells were then treated with specific primary antibodies overnight at 4°C (Table 2). On the subsequent day, after washing twice with PBS, the cells were treated with a specific secondary antibody (Table 2) and then counterstained with DAPI (4′,6‐diamidino‐2‐phenylindole) for 5 min (0.3 μg/mL) (Sigma, USA) for nuclear observation. Image analysis was performed by observing the stained cells using a laser scanning confocal microscope (Olympus, FV1200, Bio‐Health Materials Core‐Facility, Jeju National University).

### 2.7 Gene ontology (GO) analysis

GO analysis was performed to identify the biological functions of the *MyoD*, *Pax7*, *MyBPH*, *Myf5* and *Myf6* genes, using the *Sus scrofa* genomic dataset (http://asia.ensembl.org/Sus_scrofa/Info/Index) (Hubbard et al., 2002). The specific characteristics of genes related to biological function were subsequently investigated, with the analysis performed using the ToppCluster program (Chen et al., 2009; Kaimal et al., 2010).

### 2.8 Statistical analysis

All statistical analyses were performed using IBM SPSS Statistics 24 software. Quantitative RT‐PCR and protein expression analysis data were analysed using analysis of variance (ANOVA) with a two‐tailed Student's *t*‐test. The results are expressed as the mean ± standard error. Significance was accepted at the 0.05 level of probability (*p* < .05).

## 3 RESULTS

### 3.1 Differences in MRF mRNA and protein levels between Berkshire and JNPs

Quantitative RT‐PCR was performed to determine the relative transcription levels of the *MyoD*, *Pax7*, *MyBPH*, *Myf5* and *Myf6* genes. The *MyoD* gene showed higher transcript levels in piglets and adult Berkshire pigs than in JNPs (Figure 1a, *p* < .05), while *Pax7* gene showed higher transcription levels in adult Berkshire pigs than in JNPs (Figure 1b, *p* < .01), with no significant difference between piglets. The protein expression levels were consistent with the mRNA level of the MRF genes. The expression of MyoD and Pax7 was higher in 1‐day‐old and adult Berkshire pigs than in JNPs (Figure 2a,b and c; *p* < .05 for 1‐day‐old piglets and *p* < .01 for adult pigs). Interestingly, the transcription and protein levels of MyBPH were opposite to those of MyoD and Pax7; the *MyBPH* gene showed higher transcript levels in JNPs than in Berkshire pigs in both piglets and adults (Figure 1e *p *< .05), while the protein levels of MyBPH were much higher in JNPs than in adult Berkshire pigs (Figure 2a and f *p* < .001). The *MyBPH* gene and protein levels were similar in expression in piglets and adult pigs of the Berkshire breed. For the *Myf5* and *Myf6* genes, there were no significant differences in the expression levels between the piglets and adult pigs, or between Berkshire pigs and JNPs (Figure 1c and d). Inconsistent with the mRNA levels of *Myf5* and *Myf6*, the protein levels of Myf6 and Myf5 were not significantly different between the Berkshire and JNPs (Figure 2a, d, and e).

**FIGURE 1:** Transcription levels of MRFs. Quantitative reverse transcription‐polymerase chain reaction (qRT‐PCR) analysis was performed in Berkshire and Jeju native pigs (JNP). The expression levels of *MyoD* (a), *Pax7* (b), *Myf5* (c), *Myf6* (d) and *MyBPH* (e), normalized against *β‐actin* were represented. Values were presented as mean ± standard error of mean (s.e.m.) (*p < .05 and **p < .01; two‐tailed *t*‐test). JNP: Jeju native pig

**FIGURE 2:** Protein levels of myogenic regulatory factors (MRFs). The protein levels of MyoD, Pax7, Myf5, Myf6 and MyBPH were analysed by western blotting using the *longissimus dorsi* muscles of 1‐day‐old piglets and adult pigs of Berkshire and JNPs (a). Protein levels were normalized to β‐actin, and relative intensity of MyoD (b), Pax7 (c), Myf5 (d), Myf6 (e) and MyBPH (f) are represented. Values are presented as mean ± standard error of mean (s.e.m.) (*p < .05, **p < .01 and ***p < .001; two‐tailed *t*‐test). JNP: Jeju native pig

### 3.2 GO analysis of biological processes of MRFS

GO analysis of the biological processes of muscle‐related genes demonstrated how multiple genes are involved in determining the pig phenotype (Figure 3). *MyoD*, *Myf5* and *Myf6* play vital roles in the maturation of skeletal muscle fibrin and postnatal muscle‐related cells. In addition, these genes are widely involved in muscle tissue morphogenesis, muscle organ development, and muscle tissue development.

**FIGURE 3:** Cluster analysis of myogenic regulatory factors (MRFs). The dissected genes are Gene Ontology (GO) biological analysis processes shared by the MRFs in the *longissimus dorsi* muscles of Berkshire pigs and JNPs. An abstract network shows the biological pathways enriched with the cluster of MRFs specific to the *longissimus dorsi* muscle

## 4 Expression of myogenesis‐related genes through immunocytochemical analysis

The transcription levels of *MyoD* and *Pax7* were significantly higher in adult Berkshire pigs than in the piglets of this breed, whereas no significant differences were detected between adult pigs and piglets of JNPs (Figure 1a and b). To identify the localization of MyoD and Pax7, we performed immunocytochemistry on C2C12 mouse myoblast cells. Co‐expression of MyoD and Pax7 in myoblast C2C12 cells was observed, although the signal intensity was low (Figure 4). After proliferation, the activated satellite cells differentiated into myotubes or form new myotubes (Patruno et al., 2008). Our results show that the co‐expression of MyoD and Pax7 was high in activated satellite cells in myotubes formed from C2C12 cells. (Figure 5).

**FIGURE 4:** Expression of MyoD and Pax7 in C2C12 mouse myoblasts. C2C12 mouse myoblast cells showed co‐expression of *MyoD* and *Pax7*. Cells were immuno‐stained with primary antibodies against MyoD and Pax7. DAPI nuclear staining in represented in (a), and co‐expression of MyoD (green) and Pax‐7 (pink) are shown in (b). Scale bar: 10 μm

**FIGURE 5:** The expression of MyoD and Pax7 in myotube formed C2C12 cells. The cultured C2C12 myoblast cells were differentiating and myotube formation was confirmed by the observed multi‐nucleus formation in the myotube. The cells show green signals of the conjugated antibody for MyoD (a), blue signals of the conjugated antibody for Pax7 (b). The images were merged, and the co‐expression of MyoD and Pax7 is shown in the myotube‐formed C2C12 cells (c). Scale bar: 20 μm

## 5 DISCUSSION

Improving body growth and meat quality is the main aim of breeding strategies. Although JNPs have excellent meat quality, they have a slower body growth rate than the Western species, and thus pose a challenge for breeders. Therefore, many breeders seek to improve the meat and growth characteristics of JNPs. In this study, we performed comparison studies of muscle regulatory transcription factors such as MyoD, Pax7, Myf5, Myf6 and MyBPH in Berkshire pigs and JNPs (Olguín & Pisconti, 2012). MyoD is well expressed in myoblasts and myocytes during myogenesis (Rudnicki et al., 2008), triggering the conversion of many differentiated cell types into muscle (Weintraub et al., 1991). Specifically, *Pax7* and *MyoD* are involved in satellite cell differentiation (Carnes & Pins, 2020). Pietrain pigs are classified as a highly muscular breed, which is associated with the high expression of *MyoD*, *Pax7*, and more active satellite stem cells (Ropka‐Molik et al., 2011). Therefore, researchers consider that *MyoD* and *Pax7* play a significant role in muscle growth and development. Muscle mass growth in adult pigs is associated with satellite stem cells, and *Pax7* plays a critical role in regulating satellite cells; for example, during self‐renewal in the skeletal muscle (Ishido et al., 2009). This result was consistent with those of the present study; we found that Berkshire pigs showed higher expression levels of *MyoD* and *Pax7* than JNPs (Figure 1a and b; Figure 2a, b, and c). The myogenic factor *Myf5* and *Myf6* genes regulate the early stage of muscle development (Maak et al., 2006). These genes were expressed at sustained levels in postnatal fully grown muscle fibres (Weintraub et al., 1991) and are involved in the differentiation and maturation of myotubes (Wyszyńska‐Koko & Kurył, 2004). Therefore, we often consider them as candidate genes for muscle growth‐related traits in pigs. However, the expression of *Myf5* and *Myf6* did not differ between Berkshire pigs and JNPs (Figure 1c and d; Figure 2a, d, and e). These results are consistent with previous results, which show that *Myf5* or *Myf6* knockout mice have no significant differences in muscle mass (Kassar‐Duchossoy et al., 2004). The *Myf5* and *Myf6* genes were recognized to play minor roles compared to *MyoD* or *Pax7* (Carmo et al., 2005). Collectively, the present study demonstrates that *MyoD* and *Pax7* are closely associated with myogenesis and myocyte differentiation.

In this study, the ToppCluster method was used for the functional analysis of muscle‐specific genes. The analysed results are represented as a graphical network. This graphical network helps to understand the biological processes involved in the differentiation of skeletal muscle cells, the development of skeletal muscle tissue, and regeneration of skeletal muscle organs. In addition, it elucidates the role of skeletal muscle satellite cells in the development of skeletal muscle cells. The ToppCluster analysis showed that *MyoD* and *Pax7* are widely involved in the differentiation of skeletal muscle cells, proliferation of myoblasts, and skeletal muscle satellite cells (Figure 3), as shown in previous studies (Olson, 1990; Patruno et al., 2008; Ropka‐Molik et al., 2011).

Satellite cells are one of the earliest identified adult stem cells and have been reported to play an essential role in muscle regeneration, growth, and muscle cell hypertrophy (Siegel et al., 2011). Previous studies have shown that while quiescent satellite cells express only *Pax7*, the activated satellite cells co‐expressed *Pax7* with *MyoD* (Mesires & Doumit, 2002; Patruno et al., 2008). These results are consistent with the results of our myogenesis assay using C2C12 cells, where *MyoD* and *Pax7* were more highly co‐expressed in myotubes formed from C2C12 cells (Figure 5) than in myocytes (Figure 4). *Pax7* is a candidate gene that induces the self‐renewal of satellite cells and actively participates in muscle growth during the postnatal growth process (Patruno et al., 2008). In addition, activated satellite cells become inactive without *MyoD* expression (Zammit et al., 2006). The regulation of MyoD activity by the *Pax7* gene might affect muscle formation (Olguín & Pisconti, 2012). Moreover, the overall loss of muscle and decreased expression of *MyoD* were observed in *Pax7* knockout mice (von Maltzahn et al., 2013; Patruno et al., 2008). The physiological role of *Pax7* in satellite cells has also been reported as potentially influencing early postnatal growth in pigs (Patruno et al., 2008). These studies suggest that the low levels of *Pax7* and *MyoD* gene expression in JNPs may be the reason for low muscle mass and growth.

Myosin‐binding protein H (MyBPH) was first identified as a crucial myofibrillar constituent of vertebrate skeletal muscle (Gilbert et al., 1999). Skeletal muscle consists of multi‐nucleated muscle fibres comprising a bundle of elongated myofibrils (Boland et al., 2018). *MyBPH* encodes a significant component of the myosin protein in skeletal muscle, which is found in the myosin head in the Z region of the striated muscle segment. Myofibrils consist of thin and thick filaments, which contain actin and myosin (Klont et al., 1998; Zhang, 2009). Myosin, a thick filament, is a major protein that affects muscle fibre morphology. The muscle fibre type is responsible for the water content, muscle texture, colour, flavour and meat quality, as well as nutritive value (Boland et al., 2018; Sodhi et al., 2014). The results of the present study suggest that a high expression level of *MyBPH* in JNPs is crucial for determining meat quality in pigs.

## 6 CONCLUSION

In this study, we identified *MyoD* and *Pax7* as potential candidate genes for determining skeletal muscle mass in the Berkshire breed, whereas the *MyBPH* gene is involved in meat quality in JNPs (Figure 6). Although further confirmation studies are needed to elucidate the relationship between the *MyoD*, *Pax7* and *MyBPH* genes and their regulators in other breeds, the results of the present study may help to explain the genetic basis for skeletal muscle mass and meat quality in JNPs. This genetic information can assist the breeders to develop strategies for improving growth performance and meat quality.

**FIGURE 6:** Proposed model of myogenesis mechanisms for muscle mass and meat quality in Berkshire and Jeju native pigs. High expression of MyoD and Pax7 are strictly relative to muscle mass with the activation of satellite cells in the Berkshire breed, whereas high expression of MyBPH is involved in meat quality in the JNP breed

## 7 ETHICS STATEMENT

The authors confirm that the ethical policies of the journal, as noted on the journal's author guidelines page, have been adhered to and the appropriate ethical review committee approval has been received. The US National Research Council's guidelines for the Care and Use of Laboratory Animals were followed.

## CONFLICT OF INTEREST

The authors declare no competing financial interests.

## AUTHOR CONTRIBUTION

Kyoungho Kim: Data curation; Formal analysis; Writing‐original draft. Dahye Kim: Data curation; Methodology; Validation. Yunhui Min: Data curation; Formal analysis; Methodology. **DongKee Jeong:** Methodology; Resources; Software. **Youngok Son:** Funding acquisition; Supervision; Writing‐review & editing. **Kyoungtag Do:** Conceptualization; Investigation; Project administration; Supervision.

### Peer Review

The peer review history for this article is available at https://publons.com/publon/10.1002/vms3.418.
